# Management of Patients with Cervicofacial Edema and Paresthesia during Perioperative Period of Transoral Endoscopic Thyroidectomy

**DOI:** 10.1155/2022/4775264

**Published:** 2022-09-28

**Authors:** Xia Yang, Jian Guo Zhao, Mengting Liu, Shan Wang, Li Wang

**Affiliations:** ^1^Department of Thyroid and Breast Surgery, Wuhan Number 1 Hospital, Tongji Medical College, Huazhong University of Science and Technology, China; ^2^Department of Nursing, Wuhan Number 1 Hospital, Tongji Medical College, Huazhong University of Science and Technology, China

## Abstract

**Objective:**

To analyze the clinical intervention effect of transoral endoscopic thyroidectomy on the neck and face during perioperative period.

**Method:**

From January 2019 to January 2020, 60 patients included in this study were randomly divided into observation group and control group according to the ratio of 1 : 1, with 30 cases in each group. Both groups underwent rapid surgical intervention during the perioperative period. The patients in the observation group received neck and face management. The degree of jaw swelling, the degree of facial microexpression completion, and the changes in jaw and neck sensation were compared between the two groups.

**Results:**

There was no significant difference in neck and face swelling, pain, facial microexpression, and feeling between the two groups before operation. Patients with facial I/II swelling degree in the observation group were significantly more than in the control group, and the patients with III swelling degree were less than in the control group. There was significant difference for facial swelling between the two groups in the three intervention periods after the operation, and the difference was statistically significant (*P* < 0.05). The scores of facial microexpression in the observation group were higher than those in the control group during the three postoperative intervention periods, with statistical significance (*P* < 0.05). There was no significant difference in the pain score of the first day after surgery between the two groups (*P* = 0.298). In the other two postoperative intervention periods, the pain score of the observation group was lower than that of the control group, with a statistically significant difference, and the difference was statistically significant (*P* < 0.05). The threshold of chin and neck sensory pressure in the two groups was statistically significant (*P* < 0.05) except that the “cheek in area 4” (*P* = 0.290).

**Conclusion:**

The results showed that these interventions, such as the elevation of bed after operation, 24-hour intermittent cryotherapy, ice cubes in mouth, and the “meter” functional training, have good clinical effects on the symptoms of facial swelling and abnormal sensation of neck and face. It can accelerate the speed of edema dissipation, improve the patients' postoperative comfort, and improve the satisfaction and quality of life of patients with the effect of surgery and beauty.

## 1. Introduction

The incidence of thyroid diseases has been increasing in recent years, and timely and good treatment is the key to alleviate adverse symptoms [1]. Traditional thyroid surgery is mature and safe, but it will have a great impact on the maxillofacial aesthetics of patients [2]. With the progress of medical technology, the deepening of ESAR, and improvement of patients' aesthetics requirements, the oral endoscopic thyroidectomy has developed rapidly due to its advantages such as hidden scar, no wound on the body surface, and quick healing, which meets people's pursuit of minimally invasive effect and the aesthetics requirements, and has gradually become one of the routine operations in thyroid and breast surgery [2–4].

The corresponding complications of the new operation are different from other operations. Clinical practice found that oral endoscopic thyroidectomy compared with the traditions is prone to submandibular ecchymosis, mental nerve injury, facial muscle injury, and other complications affecting the lower lip and mandible motor sensory abnormalities. At present, reports of oral endoscopic thyroidectomy in China are gradually increasing, but there is little attention to the complications related to physical and psychological comfort caused by short-term decrease in facial beauty and paresthesia after surgery and no comprehensive clinical intervention measures. However, relevant studies [5] have shown that due to the particularity of the operation and physical structure of the surgical incision, postoperative tissue edema is prone to occur.

Therefore, it is urgent to strengthen the neck and face management of perioperative transoral endoscopic thyroid patients in order to reduce postoperative psychological pressure of patients, improve satisfaction with cosmetic effect and quality of life, and provide reference for later treatment. Reactive swelling is currently considered to be traumatic swelling caused by surgery, which usually occurs 2~3 days after surgery [6], resulting in facial swelling, pain, numbness, and so on. It is easy to cause anxiety and reduce the patients' satisfaction with cosmetic effect and quality of life. In recent years, our hospital has carried out more than 200 sets of oral thyroid surgery. The purpose of this study is to objectively evaluate the facial edema and skin sensation of patients after oral endoscopic thyroidectomy based on the Semmes-Weinstein test theory, combined with the related measuring instruments and evaluation tools, so as to provide clinical reference for the prevention and nursing of postoperative edema, pain, facial microexpression damage, and other complications. Now, the following report is made.

## 2. Materials and Methods

### 2.1. Patients

60 patients were enrolled in our study from January 2019 to January 2020 and were randomized into observation group and control group in 1 : 1 ratio, with 30 cases in each group. Any public report related to the results of this study will not disclose the patient's personal identity, and the patient's personal data will be strictly confidential. All patients underwent thyroid function test, thyroid ultrasonography, enhanced thyroid CT, and other routine examinations during preoperative and hospitalization. The associated surgical risks were fully passaged to the patient, respecting the patient's autonomy. There was no significant difference between the two groups in age, gender, BMI, nature of lesion, tumor diameter, and weight of resected tumor (*P* > 0.05), and the results are shown in Table 1. The qualifications of surgeons and nurses in the two groups were the same. This study was in line with the Declaration of Helsinki. Informed consent was signed before the study, and patients voluntarily participated in this study.

### 2.2. Inclusion and Excluding Criteria

The surgical indications and contraindications of patients were referred to “Expert Consensus on Endoscopic Thyroidectomy Via Oral Vestibular Approach (2018)” [7]. Inclusion criteria are as follows: (1) benign thyroid tumor ≤ 5 cm; (2) ≤1 cm thyroid micropapillary carcinoma with no evidence of metastasis; (3) the lesion was unilateral tumor by thyroid ultrasonography; and (4) patients have the willingness for cosmetic surgery. Exclusion criteria are as follows: (1) history of jaw and neck surgery; (2) severe heart, brain, lung, kidney, and other diseases that affect the safety of surgery; (3) thyroid tumors are located in the upper pole of the thyroid; and (4) a history of severe cervical spondylosis.

### 2.3. Surgical Methods

All 60 patients used mouthwash to clean their mouths before operation, took the supine position with the neck hyperextension, and intubated the trachea through the mouth for general anesthesia. The cervical white line was incised, and the thyroid gland was exposed. Unilateral lobotomy with (or without) ipsilateral central lymph node dissection was performed, oral vestibular mucosa was sutured with absorbable suture [7], and the specimens were sent to the department of pathology for examination. During the operation, three incisions (1.5 cm, 5 mm, and 5 mm) were made through the oral vestibule, and the endoscope and instruments were placed from the oral vestibule to reach the thyroid region. The subcutaneous tissue was separated by ultrasonic scalpel, and the operation space was established.

### 2.4. Study Design

#### 2.4.1. Fast Track Surgery

All patients were given clinical intervention of fast track surgery.

*(1) Preoperative*. (A) Comprehensive assessment of the patient's basic diseases and physical conditions was conducted. For example, patients with lung diseases or smokers should master effective method of coughing, and aerosol inhalation treatment should be performed when necessary. (B) Patients with hypertension and diabetes need to follow the doctor's advice and regulate the disease with rational drug use and diet guidance. (C) According to the patient's individual situation, one-to-one health education was carried out to introduce the operating room environment, intraoperative cooperation methods, and relevant matters needing attention, and emphasizing the advantages and methods of the concept of ERAS. (D) The skin and oral were cleaned before surgery. Gargling with oral cleaning solution and rinsing three times a day were made by our hospital. Teeth were cleaned if necessary. (E) Oral administration of 5% glucose 100 ml from the morning of the operation day was done. (F) Starting from the day of admission, surgical posture training was performed, including neck relaxation exercise, neck hyperextension training, deep breathing, and balloon blowing training, so as to improve the tolerance of anesthesia and reduce the risk of anesthesia. (G) The patients' psychological changes were dynamically grasp, psychological counseling was timely conducted, and successful treatment cases were explained to patients, to improve their confidence and eliminate anxiety and fear.

*(2) Intraoperative*. (A) The patient's vital signs and the changes in the amount of access were closely observed. (B) Keep the temperature and humidity in the operating room appropriate to reduce the unavoidable exposure during the operation. (C) The operator should move gently and follow the principle of sterility.

*(3) Postoperative*. (A) After the operation, the patients returned to the ward and were properly placed. The patients who were not awake after anesthesia went to the pillow and lay on their back, with their head tilted to one side. Vital signs were monitored, and special attention was paid to breathing and wound conditions. The respiratory tract was kept unobstructed and low flow oxygen inhalation was given. (B) Pressure bandaging under jaw was applied on the1st day after operation to reduce local edema. If the swelling was alleviated, the time of the head cover could be reduced. (C) If necessary, aerosol inhalation should be performed as instructed by the doctor to reduce respiratory edema and prevent infection. (D) Instruct the patients to pay attention to the protection of the operation area during activities and coughing. (E) If there was no discomfort for 6 h after surgery, the patient could take a semireclining and prevent the neck violent activity. If the vital signs were stable and the anesthesia was fully awake, patients can drink a small amount of water. If there was no other discomfort, liquid diet could be given. After 24 hours of operation, you can gradually transition to semi liquid, soft food, and common food and gargle with mouthwash before and after eating. (F) After anesthesia, turning over and stretching of limbs can be carried out on the bed, and in the first day after operation, voice training can be carried out in the early stage.

*(4) Discharge Guidance*. Patients received discharge and dietary guidance [8], and outpatient follow-up was conducted one week after surgery.

#### 2.4.2. Cervicofacial Interventions

The observation group was given cervicofacial interventions on the basis of the control group after operation:

1. After the operation, the patient returned to the ward and was given ice compress on the operation site according to the doctor's advice. The cold treatment time was 24 hours, no more than 30 minutes each time. During this period, it should be applied after an interval of 30 minutes. The purpose is to make local vasoconstriction, reduce capillary permeability, and reduce local congestion and pain caused by tissue swelling oppressive nerve endings. It was wrapped in disposable sealing bags when putting ice, taken care to sanitize the isolation principle. During cryotherapy, the local skin condition and skin color of the patients should be observed to prevent frostbite. Check the ice bag for water leakage, listen to the complaints of the patients, and stop the cold treatment immediately if there is any abnormality
2. At 2 h postoperatively, the patient's consciousness recovered and the bedside could be raised by 5-10° without discomfort. In the later stage, the patient's bedside should be raised step by step to maintain 30°, 60° of semidecumbent position, and 90° of the sitting position, so as to facilitate smooth incision drainage [9]
3. After the patient is fully conscious (2 h postoperatively), the nurse wears film gloves to give an ice block to the patient to hold it in the mouth. The ice is a sphere with a radius of 1 cm and is placed at the front of the patient's tongue tip. One piece at a time was placed in the front of tongue tip and slowly swallowed in patients with conscious state if no discomfort, every 30 min to give a piece, within 6 h; the purpose was to reduce the patients with jaw tissue swelling and pain. If there were uncomfortable symptoms such as choking, let the patient's thumb web press the operation area to cough effectively
4. Postoperative rehabilitation: at 3 days postoperatively, “meter” rehabilitation training could be started to prevent tissue scar contracture and promote blood circulation in the neck. Postoperative rehabilitation should be carried out gradually, and the actions should be slow and gentle. Avoid food of spicy and easy to plug teeth, and gargle with water after eating. Come to the hospital for reexamination one week after surgery

### 2.5. Evaluation Index

1. The soft ruler with a standard scale was used to evaluate patients' facial swelling by the Perez-Gonzalez direct measurement color Doppler ultrasound
2. VAS was used to evaluate patients' pain of the operation side. A self-made scale was used to evaluate to evaluate the facial microexpressions, including toot mouth, grin mouth, lower lip extension, and chin muscle contraction; VAS was used to evaluate the pain of the surgical site. Draw a 10 cm horizontal line on the paper, and the two ends indicated “painless” (0) and “severe pain” (10), respectively. According to the degree of feelings, the patient drew a point on the straight line which is consistent with the intensity of feeling, and the distance from the “painless” end to the mark is the feeling score. Generally, it was repeated twice, and the average value was taken. The scores were evaluated preoperatively, 1 day, 3 days, and 1 week after surgery
3. Sensory changes in the chin and neck were assessed by the Semmes-Weinstein monofilament test. Chin and neck sensory evaluation [10]: the baseline nylon monofilament test of FEI company of the United States was used to objectively evaluate the sensation of 10 areas of chin, face, and neck: area 1 (lower lip, right, and left), zone 2 (chin, right and left), zone 3 (submental), zone 4 (cheek, right, and left), zone 5 (submandibular, right, and left), and zone 6 (grade VI). The basic nylon monofilament test box is designed to fully follow the Semmes-Weinstein test theory for fine tactile examination that can measure sensations from light touch to deep pressure. The strength represented by different specifications was as follows: 2.83 = 0.07 g/mm^2^ (normal sensation), 3.61 = 0.4 g/mm^2^ (hypotactile loss), 4.31 = 2 g/mm^2^ (protective hypoesthesia), 4.56 = 4 g/mm^2^ (protective loss of sensation), and 5.07 = 10 g/mm^2^ (protective loss of sensation). The patient took the sitting position, closed his eyes, gently scratched the monofilament on the skin of the measured area, and recorded the pressure value of the lightest monofilament identified by the patient as the pressure threshold of the specified area. The measured values of the left and right areas are taken as the average

### 2.6. Data Collection and Analysis

#### 2.6.1. Evaluation of Facial Edema

The patient was in the upright position, and the mouth angle (Co), mandibular angle (Go), and soft tissue premaxillary point (Po) were selected on both sides. The body surface distances of Co-Go, Co-Po, and Go-Po were measured with a soft ruler before surgery, on the first day, the third day, and one week after operation (the average values of the left and right sides were taken), and the percentage of facial swelling was calculated according to the formula: (the measured distance on the first day, the third day and one week postoperatively − the measured distance before surgery)/the measured distance before surgery × 100%. The subcutaneous thickness at Po and 2 cm beside Po point was measured by color ultrasound.

*(1) Evaluation Criteria for Swelling [11]*. 0 degree means appearance is basically normal and facial swelling percentage ≤ 3%; I degrees means mild swelling appearance and facial swelling percentage > 3%and ≤ 6%; II degrees means the appearance of moderate swelling and facial swelling percentage > 6%and ≤ 12%. III degrees means appearance of severe swelling, local skin, and facial swelling percentage > 12%.

*(2) Facial Microexpression Evaluation*. Self-made facial microexpression questionnaire was adopted, including pout, grin, lower lip extension, and chin muscle contraction. “Fully capable” was scored as “2,” “partially capable” was scored as “1,” and “not able” was scored as “0”; the facial microexpression scores of patients in four study periods were compared (Figures 1 and 2).

### 2.7. Statistical Analysis

The IBMSPSS24.0 software was applied for statistical analysis. The measurement data were expressed by mean ± standard deviation. The counting data were expressed by frequency or rate. *t*-test was used when measurement data obey normal distribution, and rank sum test was used when it did not obey normal distribution. *χ*^2^ test was used to compare the classified counting data. Repeated measurement data were analyzed by repeated measurement analysis of variance. Main effect test results were used when there was no interaction, and simple effect analysis was carried out when there was interaction. *P* < 0.05 indicated that the difference between groups is statistically significant.

## 3. Results

1. Comparison of the degree of swelling between the two groups showed that there was no significant difference before surgery (*P* > 0.05). After intervention, there were statistically significant differences in the degree of swelling on the first day, the third day, and the week after surgery, and the difference was statistically significant (*P* < 0.05); results are shown in Table 2

(2) Preoperative VAS and facial microexpression score of the two groups were all within the normal range and were not comparable (*P* > 0.05). The VAS of the two groups was not statistically significant except “the 1st day after surgery” (*P* = 0.298), and the other two postoperative intervention periods were statistically significant. The scores of facial microexpression in the observation group were all higher than those in the control group during the 3 postoperative intervention periods, and the difference was statistically significant (*P* < 0.05), as shown in Table 3

(3) The preoperative pressure threshold values of chin and neck in the two groups were all within the normal sensory range and were not comparable. Postoperatively, except for the “cheek in area 4” data, which was not statistically significant (*P* > 0.05), and the difference was statistically significant (*P* < 0.05) at the time of postoperative intervention, which was statistically significant (see Table 4 for details)

## 4. Discussion

In this study, we found that the incision of patients undergoing endoscopic oral thyroidectomy was hidden, which brought some difficulties to the observation and nursing of postoperative incision swelling and bleeding. According to the anatomy of the mandible, oral vestibular incision may cause mental nerve injury and facial expression muscle injury, which has a certain impact on the motor and sensory function of the lower lip and mandible [12, 13]. It was reported that the lesions of the mental nerve were about 0.7%~33.3% [12, 14]. This study enrolled 60 patients with oral endoscopic thyroid surgery according to the standards of aspiration and drainage, to explore postoperative intervention measures, aimed at providing clinical reference value for patients with better recovery in the later stage.

This study was carried out for one year under the standard of admission and exclusion. Through setting up the control group and the observation group, and taking the corresponding clinical intervention, it was found that all patients in the study had swelling of mandible and neck, abnormal sensation, facial microexpression damage, and pain on the 1st day after operation, which may be caused by too much chin muscle transection during the central incision and chin muscle tearing caused by operation leverage [15]. The neck incision is hidden in the oral vestibule by oral endoscopic thyroidectomy to achieve the purpose of neck beauty and improve patients' satisfaction with the beauty effect. Our jaw and lower lip not only have the same aesthetic function as the neck skin but also have important social functions in daily life [15]. Serious swelling of patients in postoperative may lead to appearance of psychological disorder such as mouth restriction and self-image disorder, which may affect the work, life, and interpersonal communication, resulting in the decline of patients' quality of life. However, with the management of effective interventions and the extension of postoperative time, the degree of discomfort decline and recovery in the observation group was better than that in the observation group. Except for “VAS” and “cheek in the 4th zone” on the 1st day after operation, the other data of the two groups were statistically significant (*P* < 0.05), which may be related to the body stress reaction, surgical site, and incision.

Giving ice to patients after operation can effectively reduce the patient's oral temperature, the proliferation of oral bacteria, and mandibular edema. At the same time, melting ice water is slowly swallowed by patients, which is conducive to improving the comfort of patients. Therefore, keen observation and serious sense of responsibility are the keys to complete clinical work and reduce complications. Interval cryotherapy within 24 hours after surgery can slow down local blood flow, help blood clotting and control bleeding, and reduce pain caused by tissue swelling. Postoperative patients are prone to lower lip and jaw swelling, combined with high oral temperature and preoperative water prohibition. The proper and gradual elevation of the head of the bed and the cryotherapy can safely and effectively drain and accelerate the speed of facial edema dissipation, which is similar to the research results of Yuping et al. [9]. Meanwhile, according to the relevant results, it is safe to treat nerve injury by endoscopic thyroidectomy, which is the same as KYung [11].

Relevant data [16, 17] showed that continuous ice compress can reduce the sensitivity of local nerve endings and cells, thus increasing the pain threshold or shortening the pain time. Enwemeka et al. [18] found that ice compress therapy can reduce the temperature of tissue 2 cm below the skin and found that there is blood exchange between deep and shallow tissues, which explains that ice compress therapy can effectively reduce swelling and pain of local tissues. Swenson et al. [19] considered that the difference of the curative effect of ice compress lies in the difference of using method through applying ice compress to soft tissue trauma in the early stage of sports medicine. Although it is effective for patients to reduce swelling, if continuous ice compress method is adopted and ice compress medium is replaced, whether the speed of patients' swelling is faster than intermittent ice compress therapy needs further study [20–24].

Process and behavioral outcomes are just one way to measure impact. Results related to postoperative quality of life and patient satisfaction should be considered [25–29]. Similarly, the feedback and opinions of medical staff are equally important. These should be the themes of future research. The limitation of this study lies in the lack of follow-up of patients after discharge. In the next study, we should extend the study time and strengthen the intervention of patients' continuing care, so as to quantitatively evaluate the postoperative quality of life of patients. This study still has some shortcomings. Firstly, the quality of this study is limited due to the small sample size we included in the study. Secondly, this research is a single-center study and our findings are subject to some degree of bias. Therefore, our results may differ from those of large-scale multicenter studies from other academic institutes. This research is still clinically significant, and further in-depth investigations will be carried out in the future.

## 5. Conclusion

Intervention management of cervicofacial edema and paresthesia during perioperative period of oral endoscopic thyroidectomy can effectively reduce postoperative facial edema, accelerate the dissipation of swelling, improve postoperative sensory comfort, and improve the satisfaction of patients with surgical effect and quality of life.

## Figures and Tables

**Figure 1:** Data acquisition map.

**Figure 2:** Semmes-Weinstein sensory measurement.

**Table 1:** Patients' characteristics.

Variables	Observation group (*n* = 30)	Control group (*n* = 30)	*P*
Age (year)	39.10 ± 11.24	41.03 ± 7.93	0.445
Gender (*n*)			
Male	3	27	0.685
Female	4	26	
BMI (kg/m^2^)	20.08 ± 1.75	20.34 ± 1.75	0.573
Nature of lesion (*n*)			
Benign	23	7	0.519
Malignant	25	5	
Tumor diameter (cm)	1.78 ± 0.42	1.69 ± 0.52	0.486
Weight of resected tumor (g)	18.92 ± 1.55	18.31 ± 2.04	0.195

**Table 2:** Comparison of swelling degree between two groups before and after intervention.

Group	*n*	Intervention time															
		Pre-op				Post-op 1 day				Post-op 3 days				Post-op 1 week			
		0	I	II	III	0	I	II	III	0	I	II	III	0	I	II	III
Observation group	30	30	0	0	0	0	4	20	6	0	11	18	1	6	23	1	0
Control group	30	30	0	0	0	0	0	21	9	0	6	20	4	0	21	9	0
*Z*		0				-6.140				-2.032				-3.492			
*P*		>0.05				<0.05				0.042				<0.05			

Abbreviations: Pre-op, preoperative; Post-op, postoperative.

**Table 3:** Comparison of VAS (pain) and facial microexpression score between the two groups.

Group	*n*	Visual analogue pain score (points, *x̅*±*s*)				Facial microexpression score (points, *x̅*±*s*)			
		Pre-op	Post-op 1 day	Post-op 3 days	Post-op 1 week	Pre-op	Post-op 1 day	Post-op 3 days	Post-op 1week
Observation group	30	0.00	5.17 ± 1.56	2.37 ± 1.07	1.50 ± 1.01	8.00	1.60 ± 0.81	3.00 ± 1.08	6.47 ± 0.97
Control group	30	0.00	5.57 ± 1.38	3.17 ± 0.75	2.67 ± 1.24	8.00	1.20 ± 0.61	2.03 ± 0.96	4.90 ± 1.37
*t*		NA	-1.051	-3.366	-3.996	NA	2.154	3.652	5.098
*P*		NA	0.298	0.001	<0.05	NA	0.036	0.001	<0.05

**Table 4:** Comparison of chin and neck sensation (pressure threshold) between the two groups.

Zones	Pre-op (g/mm^2^, *x̅*±*s*)		*P*	Post-op 1 day (g/mm^2^, *x̅*±*s*)		*P*	Post-op 3 days (g/mm^2^, *x̅*±*s*)		*P*	Post-op 1week (g/mm^2^, *x̅*±*s*)		*P*
	*A* (*n* = 30)	*B* (*n* = 30)		*A* (*n* = 30)	*B* (*n* = 30)		*A* (*n* = 30)	*B* (*n* = 30)		*A* (*n* = 30)	*B* (*n* = 30)	
	*A* (*n* = 30)	*B* (*n* = 30)		*A* (*n* = 30)	*B* (*n* = 30)		*A* (*n* = 30)	*B* (*n* = 30)		*A* (*n* = 30)	*B* (*n* = 30)	
1: lower lip												
Left	0.07 ± 0.00	0.07 ± 0.00	NA	0.15 ± 0.43	0.61 ± 0.72	0.002	0.15 ± 0.14	0.27 ± 0.16	0.003	0.08 ± 0.60	0.16 ± 0.15	0.012
Right	0.07 ± 0.00	0.07 ± 0.00		0.23 ± 0.37	0.74 ± 0.79	0.003	0.15 ± 0.14	0.27 ± 0.16	0.003	0.08 ± 0.60	0.16 ± 0.15	0.012
2: chin												
Left	0.07 ± 0.00	0.07 ± 0.00		0.22 ± 0.37	0.67 ± 0.76	0.005	0.14 ± 0.13	0.24 ± 0.17	0.007	0.08 ± 0.60	0.15 ± 0.14	0.024
Right	0.07 ± 0.00	0.07 ± 0.00		0.22 ± 0.37	0.67 ± 0.76	0.005	0.14 ± 0.13	0.24 ± 0.17	0.007	0.08 ± 0.60	0.15 ± 0.14	0.024
3: below the chin	0.07 ± 0.00	0.07 ± 0.00		0.38 ± 0.57	0.75 ± 0.78	0.042	0.15 ± 1.14	0.28 ± 0.16	0.001	0.07 ± 0.00	0.14 ± 0.13	0.012
4: cheek												
Left	0.07 ± 0.00	0.07 ± 0.00		0.20 ± 0.17	0.25 ± 0.17	0.290	0.11 ± 0.11	0.18 ± 0.16	0.069	0.10 ± 0.10	0.17 ± 0.15	0.055
Right	0.07 ± 0.00	0.07 ± 0.00		0.20 ± 0.17	0.25 ± 0.17	0.290	0.11 ± 0.11	0.18 ± 0.16	0.069	0.10 ± 0.10	0.17 ± 0.15	0.055
5: submandibular												
Left	0.07 ± 0.00	0.07 ± 0.00		0.25 ± 0.17	0.49 ± 0.62	0.044	0.13 ± 0.13	0.21 ± 0.17	0.024	0.07 ± 0.00	0.14 ± 0.13	0.013
Right	0.07 ± 0.00	0.07 ± 0.00		0.25 ± 0.17	0.50 ± 0.62	0.034	0.13 ± 0.13	0.21 ± 0.17	0.024	0.07 ± 0.00	0.14 ± 0.13	0.013
6: neck	0.07 ± 0.00	0.07 ± 0.00		0.29 ± 0.36	0.67 ± 0.67	0.050	0.14 ± 0.13	0.26 ± 0.17	0.003	0.08 ± 0.60	0.15 ± 0.14	0.027

Abbreviations: A: observation group; B: control group.

## Data Availability

The datasets used and analyzed during the current study are available from the corresponding author upon reasonable request.
